The article "Advantage of Species Diversification to Facilitate Sustainable Development of Aquaculture Sector" was retracted in 2022. Reasons: plagiarism; overlap with other authors' work.

# Advantage of Species Diversification to Facilitate Sustainable Development of Aquaculture Sector

**DOI:** 10.3390/biology11030368

**Published:** 2022-02-25

**Authors:** Dae-Young Kim, Surendra Krushna Shinde, Avinash Ashok Kadam, Rijuta Ganesh Saratale, Ganesh Dattatraya Saratale, Manu Kumar, Asad Syed, Ali H. Bahkali, Gajanan Sampatrao Ghodake

**Affiliations:** 1 Department of Biological and Environmental Science, College of Life Science and Biotechnology, Dongguk University-Seoul, 32 Dongguk-ro, Ilsandong-gu, Goyang-si 10326, Gyeonggi-do, Korea; sbpkim@dongguk.edu (D.-Y.K.); shindesurendra9@gmail.com (S.K.S.); 2 Research Institute of Biotechnology and Medical Converged Science, Dongguk University-Seoul, 32 Dongguk-ro, Ilsandong-gu, Goyang-si 10326, Gyeonggi-do, Korea; avikadam2010@gmail.com (A.A.K.); rijutaganesh@gmail.com (R.G.S.); 3 Department of Food Science and Biotechnology, College of Life Science and Biotechnology, Dongguk University-Seoul, 32 Dongguk-ro, Ilsandong-gu, Goyang-si 10326, Gyeonggi-do, Korea; gdsaratale@gmail.com; 4 Department of Life Science, College of Life Science and Biotechnology, Dongguk University-Seoul, 32 Dongguk-ro, Ilsandong-gu, Goyang-si 10326, Gyeonggi-do, Korea; manukumar007@gmail.com; 5 Department of Botany and Microbiology, College of Science, King Saud University, P.O. Box 2455, Riyadh 11451, Saudi Arabia; assyed@ksu.edu.sa (A.S.); abahkali@ksu.edu.sa (A.H.B.)

**Keywords:** integrated aquaculture, polyculture, species diversification, species compatibility, species complementarity, sustainable development

## Abstract

**Simple Summary:**

The aquaculture sector must be well-founded to undergo robust growth and sustainable development in the years ahead. Species diversity must reflect species compatibility and complementarity to manage the complexity in polyculture systems. There is a need for the implementation of innovative strategies that facilitate sustainable aquaculture development, enhance profitability, improve resilience, and support conservation and environmental protection. An aquaculture development scenario must look beyond the economic profitability and strategize aquatic food production systems to attain food and nutrition security and benefits for all stakeholders.

**Abstract:**

Intensified agrochemical-based monoculture systems worldwide are under adoption to meet the challenge of human population growth and the ever-growing global demand for food. However, this path has been opposed and criticized because it involves overexploitation of land, monoculture of few species, excessive input of agrochemicals, and adverse impacts on human health and the environment. The wide diversity among polyculture systems practiced across the globe has created confusion over the priority of a single strategy towards sustainable aquaculture development and safer products. Herein, we highlight the significance of polyculture and integrated aquaculture practices in conveying the successful transition of the aquaculture industry towards sustainable development. So far, the established thought is that the precise selection of aquatic species and a focus on compatible and complementary species combinations are supposed to facilitate rapid progress in food production with more profitability and sustainability. Therefore, the advantages of species diversification are discussed from an ecological perspective to enforce aquaculture expansion. This account asserts that a diverse range of aquaculture practices can promote synergies among farmed species, enhance system resilience, enable conservation, decrease ecological footprints, and provide social benefits such as diversified income and local food security.

The article "Advantage of Species Diversification to Facilitate Sustainable Development of Aquaculture Sector" was retracted in 2022. Reasons: plagiarism; overlap with other authors' work.

## 1. Introduction

After the 1950s, we experienced the greatest demographic upsurge [1]. This significantly accelerated demand for food and water, which is anticipated to double in near decades [2]. Excessive expansion of agricultural land and the eradication of natural habitats have been used as solutions to meet the food demand [3]. In this context, the intensification of the implementation of agricultural practices in the green revolution has been regarded as an alternative to cut the need for new land [4]. In this perspective, most of the intensive systems have been developed for farm-specific high-yield species, typically in monoculture systems, with heavy input of agrochemicals and the use of chemical fertilizers [5]. However, such practices in the agroecosystem have resulted in environmental issues, including loss of biodiversity, food-chain adulteration, and water/soil degradation, with an eventual decrease in yields in the long term [6,7]. Therefore, sustainable agroecosystems need to be achieved by developing innovative systems and sustainable practices globally to fulfill the growing food demand [8,9]. Simultaneously, sustainable aquaculture practices have substantial scope in ensuring food and nutrient security [10,11] in place of capture fishery, which causes alarming biodiversity depletion and a possible decline in natural resources [12,13].

Similarly, further development of the aquaculture sector cannot rely completely on intensive monoculture systems. Since such systems are completely dependent on factory-formulated feed and need intensive feeding, such systems are also being criticized from a human food security and environmental point of view, lower the ability to encounter competition, and pose a higher risk of disease outbreaks [14], as well as limitations to adapting to global warming [15]. Considering these alarming circumstances, polyculture in aquaculture should be widely preferred, promoted, and practiced, as its performance adds more value to an ecosystem with several ecological services, diversified production, and consumer acceptance.

The article "Advantage of Species Diversification to Facilitate Sustainable Development of Aquaculture Sector" was retracted in 2022. Reasons: plagiarism; overlap with other authors' work.

Moreover, ecological intensification is a new concept that can address the challenges of maintaining a good production level to increase the human population while protecting the environment by conserving natural resources [16]. Essentially, the blue revolution has manifested in most parts of the world; however, it will quickly fade away unless it adopts greener practices [17]. In addition to drastically decreasing the ecological footprint of aquaculture practices, a practical implementation must be achieved with social and economic goals (diversified income) [12], thereby ensuring engagement with locals [18], fair profit-sharing [19], human well-being [20], animal welfare [21], food quality [22], and development of value-added products [23]. The current composition of polyculture systems is much more diverse than before, including fish, shellfish, mollusks, crustaceans, aquatic plants, and algal species; thus, the growth of global aquaculture in a wide variety of brackish, marine, and freshwater in global settings is estimated to grow at a rapid pace [24,25].

Finfish and crustacean products are being globally traded and their overall performance and environmental functions are being increasingly improved by collective efforts, government regulations, public and private sector standards, and marketplace incentives [25]. Of all the sustainable aquaculture practices being investigated as alternatives, polyculture and integrated aquaculture systems can be potential approaches to ensure sustainability through taxa cohabitation, ecosystem functioning, and biological interactions among combined species (glossary of terms used in the manuscript is shown in Table 1) [25,26,27,28]. Culturing diverse species based on species complementarity and compatibility in a farm setting can optimize resource use, with the primary species’ waste being utilized by the other species [29,30]. Facilitating this shift from monoculture to polyculture and integrating aquaculture systems by harnessing species diversity is widely considered a fundamental agro-ecological principle to redesign sustainable aquaculture systems for the future [31,32].

This review describes potential approaches to facilitate a smooth transition from conventional aquaculture techniques to develop more sustainable aquaculture practices that support various designs and configurations, which can aid in this transition. Critical assessments of polyculture and integrated aquaculture practices, along with their merits and demerits, are still scarce in scientific literature. For that reason, we discuss the potential aquaculture approaches that involve species diversity at different spatiotemporal dynamics and enforce its sustainability. Furthermore, we investigate recent developments to ascertain real-world challenges and inform research prospects to facilitate sustainable aquaculture development.

The article "Advantage of Species Diversification to Facilitate Sustainable Development of Aquaculture Sector" was retracted in 2022. Reasons: plagiarism; overlap with other authors' work.

## 2. Species Diversification in Aquaculture: Systemic Approach for Sustainable Food Production

### 2.1. Species Compatibility: Principle of Polyculture

Polyculture is an important principle of permaculture that involves species compatibility and complementarity in the context of sustainability and environmental protection, animal welfare, and resource sharing. It can be reinforced by combined ecological aquaculture and agroecology practices [34]. A new vision for aquaculture development needs to be implemented by incorporating comprehensive planning and meticulous implementation to obtain better results in cultivated aquatic ecosystems [53,54]. Conventional polyculture approaches encourage synergies among combined species and/or other aquaculture compartments [55,56,57]. Learning from conventional wisdom can be a potential strategy in designing innovative polyculture systems and environmentally balanced aquaculture practices that can reduce the carbon footprint, improve water quality, and increase food supply [58,59]. 

Polyculture in aquaculture needs basic compatibility among combined taxa to avoid predation behavior as feasible and interspecies competition over accessible resources. Thus, such an environment ensures the well-being of aquatic life and the overall productivity of the established system. The polyculture of pelagic and benthic aquatic species is an excellent example of intrinsic species compatibility [60,61], which naturally limits interspecific competition [62,63]. Understanding changes in ecological functioning by the use of cascade effects is inadequate and, thus, further hypothesis-driven research efforts with the integrative ecological assessment are needed [64]. 

Ad libitum feeding ensures feed availability in all growth phases, which can be enforced to avoid expected interspecific competitiveness; such management systems can facilitate compatibility among farmed species [65]. Species compatibility mainly relies on two main factors: managing the cultivation environment to ensure constant availability of feed, thereby encouraging species-specific behavior, and limiting detrimental interactions among farmed species at different developmental stages [66]. For example, the farmed species could be compatible during the initial growth stage; however, due to variation in growth rates, detrimental interactions may occur in later stages, leading to predation behavior or trophic-level competition. One important study demonstrated the significance of different stocking densities and early stocking of tilapia (*Oreochromis niloticus*) following seabass (*Lates calcarifer*) and their effect on growth and survival rate without any supplementary feed provision to seabass [67]. This report claimed that the seabass–tilapia polyculture system can be an appropriate solution to address the excessive breeding issue in tilapia and sustainable production of high-value seabass fish. Compatibility among combined taxa cannot be sustained once existing species establish negative interactions or behaviors (e.g., aggression, predation, hostility) or competition over accessible resources (space, food, or shelter). These observations suggest that it is important to evaluate the species compatibility during all the developmental stages and use alternative methods to establish species compatibility during all growth stages. Likewise, there is concern for combined species’ physiological stages; certain species become incompatible due to their differences in growth rates or changing diets over time, resulting in predation behavior. Therefore, stoking densities and composition of the combined species need to refer to species traits and positive interactions. For instance, numerous studies have revealed that system performance and fish growth largely depend on stocking densities [61,62,63,64].

The article "Advantage of Species Diversification to Facilitate Sustainable Development of Aquaculture Sector" was retracted in 2022. Reasons: plagiarism; overlap with other authors' work.

There is also a need to assess potential interspecies pathogens in designing species combination and stocking density. Moreover, combining certain species may trigger spillover interspecific pathogens [68,69,70]. The risk of interspecific spillover is often concerned with introducing exotic species [71], which suggests considering indigenous species to institute species combinations in conventional polyculture systems. Alternative aquaculture practices involve developing strategies that reflect the spatial distribution of applicable combined species to eliminate negative interactions [72], such as sequential polyculture or cage-cum-pond systems [73]. Overall, a polyculture system based on species compatibility allows us to harvest diverse aquaculture products and aids in direct environmental benefits [74]. Another import approach in achieving sustainable aquaculture development is adopting better management practices by considering compatibility among combined taxa or practicing prospective polyculture systems as presented in brief (Table 2). Furthermore, in aquaculture management, the main objective should be maximizing net economic profits and social objectives to promote the aquaculture sector more progressively and sustainably [75]. 

The article "Advantage of Species Diversification to Facilitate Sustainable Development of Aquaculture Sector" was retracted in 2022. Reasons: plagiarism; overlap with other authors' work.

### 2.2. Species Complementarity: Benefits of Polyculture

Basic complementarity allows the combination of compatible species and utilization of accessible resources (i.e., feed, shelter, space) in a given aquatic environment (Table 2) [14]. Certainly, compatible species facilitie maximum use of accessible resources in a complementary manner, i.e., species-specific resource utilization positively interacts among farmed species through trophic flows and/or develops beneficial interactions, e.g., mutualism or commensalism. Some species exhibit such behaviors in given farming environments, which opens up the possibility of controlling basic to enhanced complementarity among combined species.

#### 2.2.1. Basic Complementarity

A well-known example of a conventional polyculture system using differently specialized species of the Chinese carp (Figure 1a) exhibits an aquaculture approach based on the multi-trophic principle [57]. It integrates the involvement of various species with diverse trophic niches in the same rearing environment, which mimics their synergy in their natural habitats [14]. Basic complementarity can also be successfully implemented for some other combined fish species that utilize identical trophic resources in different spatially distributed niches, as illustrated in Figure 1b [63,76]. These “mono-trophic aquaculture systems” are sometimes less favorable for maintaining ecological balance than “multi-trophic aquaculture systems” [73]. Such integrations of compatible species would also involve additional management practices and processes to ensure improved species complementarity.

#### 2.2.2. Enhanced Complementarity via Trophic Interactions

Improved species complementarity can be established based on multi-trophic interactions, which involve an integrated agri-aquaculture perspective. The organic waste of one farming system serves as a feed source for another subsystem with enhanced ecological integrity, thereby increasing the performance of the aquaculture systems [48]. At the end of the 20th century, applying integrated aquaculture practices contributed to the improvement of integrated multi-trophic aquaculture (IMTA) [88] and integrated agriculture–aquaculture (IAA) [57,89].

The IMTA concept is extremely flexible compared to the traditional polyculture system, typically integrating biota from different tropic levels [90]. The IMTA concept has recently received more attention in worldwide research since it has been successfully demonstrated as a potential approach to make aquaculture more profitable and sustainable in both land and sea settings [74]. IMTA is currently emerging as a land-based intensive tank culture system. Several strategic developments are in progress, including open-water or land-based systems, freshwater or marine systems, and the integration of several species. Indeed, the chemical and biological processes in an IMTA should be in balance. This is mostly achieved by the selection of appropriate species in the right ratio performing different ecosystem functions [91].

The article "Advantage of Species Diversification to Facilitate Sustainable Development of Aquaculture Sector" was retracted in 2022. Reasons: plagiarism; overlap with other authors' work.

Furthermore, trophic interactions in IMTA systems can be modulated using constant water flows, e.g., by linking pellet-fed shrimp or fish species in a marine offshore system with species that feed on dissolved organic or particulate matter (e.g., fish, mollusks, echinoderm species) and another fish species that feeds on inorganic content (e.g., microorganisms, macro-algae, or macrophytes) [92], as illustrated in Figure 2. IMTA near marine seashores is being extensively investigated and can, therefore, be crucially involved in establishing a modern aquaculture industry in offshore areas. Such systems also hold tremendous scope for multiple uses of offshore facilities. It can provide additional environmental benefits if safer bio-waste products are used and transformed into valuable fresh food products. IMTA systems established using an ecosystem-based approach can achieve sustainability through alternative means, particularly in intensive aquaculture systems [88]. A closed circulatory IMTA system has been reported as an appropriate model to ensure sustainable aquaculture practices because it successfully produces sea urchins, seaweed, and fish simultaneously.

The implementation of an integrated approach in aquaculture systems is mostly carried out by combining species from different trophic levels with mutual interactions, defined as the IMTA system. However, it is essential to determine the significance of the IMTA system, usually involving the implementation of diverse approaches [46,93], which can be established in terrestrial settings, seaside marine locations, and offshore settings, as well as in the Mediterranean area [94]. IMTA is a recently developed aquaculture system; therefore, several efforts are currently being made to introduce additional features into the system [59] to ensure that it is environmentally benign, ecologically efficient, profitable, and product-diversified [95], in addition to increasing food production [88] and eventually achieving commercial food production [96]. However, implementation of the IMTA system at a commercial scale has rarely been attempted; further evaluation is required to explore the possibilities of co-occurring farming systems at the landscape scale. A recent study outlined essential recommendations to implement IMTA systems and a framework of an ecosystem approach to increase the success of commercial aquaculture farms [97,98].

The article "Advantage of Species Diversification to Facilitate Sustainable Development of Aquaculture Sector" was retracted in 2022. Reasons: plagiarism; overlap with other authors' work.

IMTA systems can also be allied with modern aquaponics systems, where trophic complementarities between domestic animals and aquatic plant species are mediated by water without using soil. IMTA-based aquaponics can be established based on natural biological cycles with increased use of accessible resources [99], which involves the integration of plants, microorganisms, and fish [100]. Therefore, this system utilizes the nitrates from the nitrogen-rich waste of fish as a nutrient input for intercropping in an aquaponic system [101,102]. IMTA aquaculture systems have several advantages, including the use of aquaculture waste by secondary species, built-up ecologically sustainable aquaculture systems, improvement of water quality, elimination of biological waste residues, and financial benefit compared to monoculture rearing systems [103]. However, a deeper understanding of trophic levels, species-specific feeding habits, and living space preferences are essential to ensure less competition among species and good overall performance of IMTA and polyculture practices. Furthermore, it is a rapidly evolving science that can be expected to be more in demand, driven by the increasing population and public awareness of climate change. Nonetheless, it is essential to increase awareness about aquaculture systems’ environmental friendliness, safety, affordability, and sustainability.

IMTA systems can result in better production compared to overall aquaculture systems, owing to mutual benefits to the integrated species and enhanced ecosystem health. In IMTA, several aquatic species from different trophic levels can be carefully considered in an integrated system to promote environmental sustainability (see Figure 2), including improving overall efficiency, reducing the formation of waste, increasing productivity, and providing ecosystem services [104]. However, an often-encountered criticism of marine finfish net-pen aquaculture is that the uneaten feed and wastes pollute the bottom layer in aquaculture system typically under the pens [105], releasing nutrients that contribute to outbursts of algal bloom formation. Poorly managed intensive finfish and crustacean systems can contribute to the emergence of harmful pathogens and algal blooms, and sea urchins, shellfish, and sea cucumbers are very sensitive to toxic microalgae [106]. Thus, integrated species should be more than just biofilters; there is a need to consider organisms that convert soluble and solid nutrient discharges from the fed species and waste feed, together turning into sizable production with commercial value that is acceptable to consumers. An in situ biofiltration strategy was proposed to limit the dispersion of waste effluents from brackish water marine finfish cage aquaculture systems [107].

The article "Advantage of Species Diversification to Facilitate Sustainable Development of Aquaculture Sector" was retracted in 2022. Reasons: plagiarism; overlap with other authors' work.

The economic feasibility of polyculture is dependent directly on the involvement of the trophic complementarities of the co-combined species that maximize the use of all nutrient resources accessible in the given ecosystem [81,92]. Aquatic species from the lower trophic levels (typically invertebrates or plants) are considered to use waste byproducts such as uneaten feed and feces from the higher trophic species farmed (typically finfish) (Figure 2) as a nutrient source [108]. The lower trophic species, e.g., seaweed, shellfish, and sea cucumber, can be harvested along with the integrated fish species to provide more revenue. Furthermore, sea cucumber (*Holothuroidea* sp.) can ingest fouling debris from salmon nets and subsequently transform it into in-demand products [109], suggesting that polyculture systems potentially replace conventional products used in cleaning practices. Such species are identified as appropriate to improve economic performance via trophic levels or directly by reducing the need for excessive cleaning or controlling fouling on the net surface, thus improving culture environment and water flow [110].

Altogether, filter-feeding finfish, mollusks, and seaweeds have demonstrated their sustainable features, mainly because they do not depend on artificial aquafeed [14]; they feed on nutrients directly from the water column. However, terrestrial crops that need to form aquafeed are expected to increase in the near future as the production of crustaceans and finfish is expected to expand in freshwater and marine settings. Moreover, it was suggested that the integration of finfish and alone with bivalves does not signify an appropriate approach in reducing the negative impacts on the environment from finfish farming [111]. Finfish markets exist for several species, including red cobia (*Rachycentron canadum*), snapper (*Lutjanus campechanus*), spotted sea trout (*Cynoscion nebulosus*), red drum (*Sciaenops ocellatus*), southern flounder (*Paralichthys lethostigma*), and several other species [112]. So far, much focus has been on finfish species; however, shrimp and blue crab (*Callinectes sapidus*), are exclusively economically important opportunities.

The article "Advantage of Species Diversification to Facilitate Sustainable Development of Aquaculture Sector" was retracted in 2022. Reasons: plagiarism; overlap with other authors' work.

IMTA can be more complex when considering several co-integration strategies, including fed species (such as shrimp or finfish) accompanied by extractive species, e.g., suspension-feeding (such as oysters and mussels) and deposit-feeding (such as sea-urchins and sea-cucumbers) species, as well as macroalgae (e.g., kelps) and invertebrates, which feed on the inorganic and organic nutrients dissolved in effluents generated by the potential fed species [91]. A recent report suggested that dog conch (*Laevistrombus canarium*) ably adapts to different environmental conditions and has a high growth rate, making it a favorable IMTA species and able to be co-cultured with sea urchins and abalone in seawater or with saltwater tilapia in land-based aquaculture [113]. Moreover, the IMTA approach is most appropriate to promote a circular economy on the basis of the economic viability of integrated aquaculture species [114] like filter feeders [115], particularly shellfish or mollusks [116].

IMTA can allow other organisms in proximity to net-pens to be fed that can use such wastes as nutrients. In IMTA, kelp was successfully grown in proximity to salmon net-pens by utilizing excreted nitrogenous wastes by farmed fish, as demonstrated in an initial trial in Canada by Cooke Aquaculture [117,118]. In a recent report on innovative IMTA systems, integrated sponges, polychaetes, and macroalgae were demonstrated in an on-shore mariculture plant located in southern Italy [119]. The environmental sustainability of aquaculture can be enhanced by establishing integrated marine aquaculture systems [93,120,121]. However, to establish IMTA as an economically viable system, each of the considered components need to be marketable [122] or add some value to the system by providing ecosystem services for those extractive species [123]. Since 2009, the Center for Cooperative Aquaculture Research (CCAR) has been working on IMTA research. Their study demonstrated how to capture wastes from a halibut tank system and use them to feed marine worm beds. The worms thrived well on the waste feed and feces, thus requiring minimal feed input, as demonstrated in a recent report [124]. After seeing such developments, one can make further efforts in seeding the bottom column with a salmon net-pen with abundant sandworms; thus, it can be reared more sustainably. Other studies are needed to explore novel approaches to colonize the sediments present under the pens with sandworms. However, there is still confusion over determining any of the possible anticipated benefits using sediment chemistry [113].

Consequently, the IAA system involving enhanced complementarity among combined species can be successful by involving terrestrial agriculture and livestock animal units with aquatic food production systems, as illustrated in Figure 3. This system encourages agricultural divergence, wherein the aquaculture module usually involves semi-intensive rearing of omnivorous or herbivorous fish (e.g., tilapia species, carp species) through the integration of terrestrial-based domestic animals and crop production practices [125,126]. In IAA systems, most farmers prefer integrating fish farming predominantly with rice farms, poultry units, or pig farms [57]. More specifically, IAA systems are mainly being implemented in Southeast Asian countries, wherein freshwater fish species are integrated with the rice fields or with aquaponic vegetables and fruits using nutrient film technique-based aquaponic systems [127], and can also be integrated with domestic animals (cattle, pig, or poultry units) [55,128]. The integration of aquaculture with a broader range of farming settings is being promoted to improve food production, preserve the environment, and ensure food security in developing countries [33,129].

The article "Advantage of Species Diversification to Facilitate Sustainable Development of Aquaculture Sector" was retracted in 2022. Reasons: plagiarism; overlap with other authors' work.

IAA systems are generally family-owned farm enterprises that include three important bases: household, agriculture, and aquaculture. Such systems can potentially generate synergies between agricultural activities and aquaculture systems, ensuring efficient resource use, enhancing nutrient recycling, and increasing overall food production. The main positive interactions of the IAA system were described in a previous report [57]. It involves using animal manure as aquaculture fertilizer, agriculture by-products as a feed supplement for fish, deploying fish waste and pond residues as crop fertilizer, and using aquaculture wastewater for irrigation [130]. Other positive interactions are also possible between farm components—for instance, control of weeds and pests in rice fields by fish [131], integrated parasite management [132], and utilization of farm residues to promote the growth of periphyton algae [133].

There is always a trade-off among farming components, and more possibilities for positive interactions can become evident through comprehensive studies of implemented IAA systems. The resilience theory also needs to be applied to provide a theoretical framework and direct further investigations of IAA systems, including incorporating farm dynamics, positive interactions, and social–ecological perspectives. Future challenges facing the implementation of IAA systems need to be highlighted to ensure that aquaculture can offer diversified income sources and crucially contribute to future food production, especially compared with those of intensive aquaculture systems. However, an integrated IAA system is not a standard-size practice, particularly in marginal settings, where integration with agriculture is more challenging than increasing farm productivity [134].

The article "Advantage of Species Diversification to Facilitate Sustainable Development of Aquaculture Sector" was retracted in 2022. Reasons: plagiarism; overlap with other authors' work.

#### 2.2.3. Enhanced Complementarity via Mutualism or Commensalism

Future R&D efforts in ecological engineering are necessary to understand negative interactions such as competition, predation, and physical disturbance that determine community structures [135]; however, its role in shaping natural ecosystems needs to be investigated further [136,137]. Predation is a type of top-down control; therefore, its negative influence starts from the top of the food chain and cascades downwards to lower trophic levels [138]. A complex trophic cascade follows when most predators ultimately affect the abundance of more than two species towards lower trophic levels [139]. The mechanism of planktivorous forage fish species has also been reported, highlighting their essential role in marine food webs by linking top-down and bottom-up control [140]. Therefore, excessive fishing can ultimately impact the plankton ecosystem, and the environmental effects cascade further onto demersal fish and predatory seabirds [141]. Furthermore, opposing top-down and bottom-up effects, including a combination of species, has significance in preventing extensive shifts in community dynamics and functioning.

Aquaculture practices need sea space or land and water of adequately high quality; both are limited resources and necessary for agroecosystems. However, there is a great scope for aquaculture development for species that fall under lower trophic levels that are not limited by fishery dependency, e.g., shellfish [142]. However, the scope in the growth of aquaculture practices for predatory marine fish is very constrained but certainly possible [138]. Frid and Paramor (2012) suggested three different possibilities for the development of predatory marine fisheries: (a) improving feed conversion ratios by using sustainable feed materials, (b) increasing the supply of fishery products by implementing effective aquaculture strategies and avoiding ecological damage, and (c) employing polyculture approaches via the cultivation of species either feeding directly on the given stock or depending on the fish-feed supply chain, including filter-feeding shellfish [138].

Despite the great significance and ubiquity of commensalism and mutualism, most positive interactions remain understudied compared to detrimental interactions such as competition, aggression, and predation. Although Greek scientists noted mutualistic interactions over 2000 years ago [143], R&D activities focused on understanding positive interactions in aquaculture systems are still relatively insufficient [144,145]. Mutualistic interactions can occur when interactions among species result in reciprocal benefits. However, the consequence of such interactions may habitually shift from positive to either neutral or negative. Depending on the farming environment and community context, these unexpected mutualistic relationships can have wide consequences. In aquatic systems, mutualism is commonly supported by an ecosystem that defines foundation mutualistic species triggering energy and nutrient dynamics between and within ecosystem settings. It provides a friendly environment with mutual benefits through mechanisms wherein species can rapidly adjust to each other and ecological diversity [146].

The article "Advantage of Species Diversification to Facilitate Sustainable Development of Aquaculture Sector" was retracted in 2022. Reasons: plagiarism; overlap with other authors' work.

Herein, we highlight the impact of positive interspecies interactions, because they exist in natural ecosystems and act as central drivers of community structure and abundance mechanisms. Fostering beneficial interactions such as mutualism or commensalism among various combined species in polyculture can be a practical approach for sustainable food production compared to monoculture. An ecological process of mutualism is popularly spread for fish polyculture practices in South Asian countries. The positive relationships among *Catla*, *Labeo rohita*, and common carp species (*Cyprinus carpio*) are based on the key ecological concept called facilitation [147]. The scavenging behavior of the carp species in such a polyculture system is beneficial to the *Labeo rohita* fish through the suspension of settled nutrients in the sediments of the water columns (Figure 4a). This behavior results in a bottom-up food supply [83], which considerably enhances rice–fish production compared to monoculture aquaculture farming systems [148]. This type of bottom-up force influences several communities to prefer lower to higher trophic levels in the food chain. Polyculture based on mutualism or commensalism can also replace excessive pharmaceutical interventions and disease control treatments by facilitating positive biotic interactions among combined species [39]. For instance, Ballan wrasse (*Labrus bergylta*) cannot be an extra product to be sold for consumption, but is useful as a cleaner fish to control sea lice in Atlantic salmon (*Salmo salar*), as shown in Figure 4b, which is a type of mutualism is being increasingly used in cage-based polyculture practices [149]. Integrated pest management to control sea lice relies on the use of licensed pesticides and effective management tools, including stocking density by the single-cohort method, optimizing stock densities, and using cleaner fish in polyculture [150,151].

The article "Advantage of Species Diversification to Facilitate Sustainable Development of Aquaculture Sector" was retracted in 2022. Reasons: plagiarism; overlap with other authors' work.

Positive interactions among species such as commensalism and mutualism are also pivotal in determining community structures and functions [39]. Therefore, considering positive interactions with ecological engineering can fundamentally improve our understanding of the processes and mutualism mechanisms that organize communities [135,153]. The significance of mutualistic relationships in aquatic communities can address several concerns: (1) Widespread mutualism in ecological communities; (2) mutualism is not necessarily the same in all ecological settings (it can be adverse in another setting); (3) usually some interactions observed as antagonistic can also be mutualistic for different community and ecological settings; (4) mutualism may not be co-evolved or constantly coupled in time or space; and (5) mutualistic interactions have a significant impact on community structures and functioning [154,155]. To our understanding, positive interactions and their influence on community structures and ecosystems are mainly identified from investigations of terrestrial settings [156] and marine environments [157,158]. However, relatively few R&D activities have reported positive interactions among freshwater aquaculture systems, even though some mutualistic interactions have existed for a century.

## 3. Shrimp, Crab Polyculture

Herein, we discuss sustainability aspects of polyculture systems established for shrimp and crab farming by considering several types and common examples of positive or beneficial interactions. It is revealed that shrimp monoculture severely affects the ecosystem, and thus, integrated aquaculture practices can be a good alternative. Innovative aquaculture practices such mangrove silvo-aquaculture systems [159], rice–crab fish culture [160], intensive pond aquaculture (IPA) or organic aquaculture [161], biofloc systems [162], integrated closed recirculatory aquaculture systems (RAS) [163], water probiotics [164], and constructed wetlands represent potential in developing innovative crab–fish or shrimp polyculture technologies [165]. So far, China has made extensive efforts to encourage aquaculture production by increasing technical advances, which is the main component of Chinese aquaculture development; however, some of the existing challenges and constraints need to be addressed. Despite the considerable progress in and advantage of shrimp aquaculture systems, this sector is facing several problems, including several diseases [166], constantly decreasing prices [167], and raising environmental impact, mainly in the form of effluents [168,169]. Some approaches, including the application of probiotics [170,171], use of antibiotics [172,173], implementation of circulatory systems [174,175], bioremediation of waste effluents [176,177], and development of innovative polyculture systems with other aquatic species [178,179,180], are being recommended to avoid certain problems.

The article "Advantage of Species Diversification to Facilitate Sustainable Development of Aquaculture Sector" was retracted in 2022. Reasons: plagiarism; overlap with other authors' work.

According to the report by Bunting (2008), polyculture systems consist of combining one or more subordinate species with the main species in the aquaculture system [181]. Recently, research reports on polyculture have increased, in some cases demonstrating a cost-effective and sustainable movement for both marine and freshwater systems [179,180,182,183]. Likewise, some other reports have indicated that combining a subordinate or secondary species certainly enhances the overall performance of the main species cultivated [58,184,185,186]. Possibly, mollusk species (*Crassostrea gigas*, *Chione fructifraga*) and fish species (*Oreochromis urolepis hornorum*) combined with other fish species [179,187] have demonstrated co-culture with shrimp species, enhancing the production factors of the shrimp. However, polyculture systems are not yet widely practiced for shrimps; indeed, there is a concern for losing the shrimp harvests; the probability of pathogens, bacteria, or viruses entering the aquaculture system; and in some cases, insufficient understanding of polyculture practices and principles. The present account highlights key principles, benefits, innovative strategies, and polyculture practices of shrimp to facilitate scientific development and sustainable activity.

There is huge potential to increase overall profitability and productivity in aquaculture by adopting innovative sustainable technologies. Its large-scale production is being established [188] and is worth more than USD 10 billion in economic benefits annually [189]. Polyculture is also referred to as co-culture [190]. There are at best three common types, including direct, pond-cum-cage, and spatially sequential polyculture (Figure 5) [48,73]. A direct polyculture system is the simplest form of co-culture, and it can be performed on most farms. However, this method has certain limitations in terms of species compatibility and the rearing capacity of the system. However, there is no need for extra space, and perhaps better control over cultured species is possible in direct polyculture (Figure 5a). Some of the most significant considerations include feed requirements and the environmental conditions needed for the combined species co-cultured with the shrimp [191]. Pond-cum-cage polyculture is somewhat different from direct polyculture, as different farmed species are co-cultured in the same pond or tank (Figure 5b), but one or more of the species are reared within cage systems, thus limiting their physical contact and space with the main species farmed [192]. However, such cages require an extra financial investment, but this investment can be reduced by using some types of cages that can be assembled with inexpensive materials such as polyester or polyvinyl chloride and plastic nets. Extreme temperatures in certain regions at the peak of summer make the cage system unsuitable; otherwise, the height of the cages should be adjusted during the day and at night with optimal levels of oxygen [193].

The article "Advantage of Species Diversification to Facilitate Sustainable Development of Aquaculture Sector" was retracted in 2022. Reasons: plagiarism; overlap with other authors' work.

The spatially sequential polyculture method involves the integration of aquaculture systems, wherein main and secondary or subordinate species are farmed separately by setting adjacent units, and waste effluents flow from the shrimp system to other culture units made for secondary species (Figure 5c). In some systems, the wastewater is discharged and in others it gets recirculated [194]. The subordinate species thrives well in the target species’ effluents, feeding on the organic–inorganic matter, non-consumed feed, and some other waste nutrients. Thus, this approach can improve the overall quality of the wastewater, or the wastewater can be reclaimed for irrigation purposes and decrease the negative impact on the environment [195]. In polyculture, each species has different physiological needs or minimal competitive, antagonistic, or predator interactions; otherwise, the success of the polyculture practice within the same unit turns unlikely. Thus, such systems can be an alternative solution [194].

Two key strategies can be implemented in these types of polyculture systems. The first is mono-trophic aquaculture, wherein similar species in terms of physical and nutritional needs can be combined in the same culture system, e.g., two or more species of shrimp [196]. The other is multi-trophic aquaculture, wherein species from distinct trophic levels are considered in the aquaculture system (e.g., fish–shrimp–seaweed). It was emphasized that aquaculture could combine fed species (e.g., shrimp or finfish) with inorganic extractive species (e.g., seaweed), and finally, organic species (e.g., deposit- and suspension-feeders) cultured in proximity [92].

Some other species have good commercial value; those can be potentially good candidates with a high market value in polyculture systems—for example, sea cucumbers [197]. Similarly, tilapia is also a better candidate for polyculture with shrimp species [198], as it holds high resistance or protection against certain bacterial and viral diseases [187,199,200,201], robustness to adverse conditions [202], enhanced commercial profitability [203], and different feeding habits [204]. Likewise, macroalgae *Kappaphycus alvarezii* can be integrated into shrimp polyculture and has a commercial value and is used to produce the thickening and stabilizing agent called carrageenan [205]. Several other aquatic species can also be integrated, including *Ulva clathrata*, *Gracilaria salicornia*, and duckweed (*Lemnaceae* sp.), which have been cultivated using nutrient-rich wastewater from shrimp aquaculture systems [206,207,208].

The article "Advantage of Species Diversification to Facilitate Sustainable Development of Aquaculture Sector" was retracted in 2022. Reasons: plagiarism; overlap with other authors' work.

Consequently, demand for another important crustacean-like crab is ever-growing in the international market. Crustacean culture, in general, is most profitable in terms of high commercial value [73]. Shrimp farming is known for high yield potentiality and providing higher returns to farmers [209]. Moreover, consumers often prefer organic shrimp products, which remains highly profitable [210,211] and has positive implications on the socio-economic status of stakeholders and environmental benefits [212,213]. Another important crustacean example is crab farming, which has several success stories in aquaculture development and provides a reliable source of income for rural stakeholders [214].

A native freshwater Chinese mitten crab is one of the important crustacean species for aquaculture and is widely farmed all over the eastern region of China [215,216,217]. However, despite this industry’s progress, monocultures still face several challenges and technical problems, including diseases and environmental pollution. For instance, polyculture systems of shrimp crabs have numerous benefits that could contribute to achieving less impact on the environment, enhancing production, and improving discharge effluent quality [161,179]. Shrimp–crab polyculture could achieve a reduction in inorganic nitrogen via microbial assimilation [218], as demonstrated in a recent report on microbial diversity, which was found to be significantly higher in polyculture than in monoculture systems. Furthermore, that report claimed that the shrimp polyculture system allows fatty acid biosynthesis to be enhanced more than in monoculture, in addition to the enhancement of other biological processes, including higher oxidation–reduction potential, total organic carbon, and total phosphates that can be achieved, signifying the formation of a relatively less anoxic setting.

There is a long history of polyculture practices in several Asian countries [219,220]. However, there is a lack of sufficient knowledge about the farmed species and polyculture systems as important factors that need to be considered during co-culturing crab or shrimp species with other subordinate species. This scenario raises an important issue: improving shrimp, crab, or other subordinate species polyculture practices and increasing yield. Therefore, more efforts to raise awareness of recent developments in polyculture systems are greatly recommended, particularly for the marginal and small-scale rural farmers [221]. Wan et al. revealed the importance of co-culture in aquaculture, including Chinese mitten crab (*Eriocheir sinensis*), which has several benefits in terms of productivity for local farmers [222].

The article "Advantage of Species Diversification to Facilitate Sustainable Development of Aquaculture Sector" was retracted in 2022. Reasons: plagiarism; overlap with other authors' work.

A recent study evaluated the effect of stocking densities on the phosphorus and nitrogen budget in polyculture enclosure systems for crab species (*Portunus trituberculatus*) and Pacific white shrimp [223]. That report revealed significant findings that the polyculture system developed for shrimp with crabs in appropriate densities, improving overall profitability, productivity, nutrient utilization, and environmental sustainability. Intrinsically, the potential farmers identify a need for organic practices in aquaculture that allow polyculture practices to be promoted and encourage the selection of endemic/indigenous species under either extensive or semi-intensive aquaculture systems [224]. Such systems also allow inputs of artificial ingredients to be minimized, better possibilities for genetically modified species to be found, and ecological functions essential for sustainable aquaculture development to be considered. Organic aquaculture practices need to positively and significantly influence all stakeholders to encourage the adoption of improved IPA technologies in the organic prawn–crab polyculture system. Another important report on polyculture of mud crabs with finfish revealed more profitability with sustainable diversification of brackish water farming [225]. The observation in the recent study reported by Li et al. (2014) showed that rice–crab systems have several benefits, including reductions in input costs, better profitability, and increased ecological sustainability compared to the rice monoculture systems [226].

Several other benefits, including reducing environmental impacts, enhanced yield, and improved water quality, have been documented in shrimp polyculture systems by integrating fish species, bivalve species, and seaweed as subordinate species; currently, polyculture systems are being commonly and extensively researched [163,227,228]. There is also an indication that the relationship of combined species diversity within a given environment influences different ecosystem processes, including overall productivity, nutrient decomposition, and cycling [229,230,231]. Furthermore, a polyculture system allows the production of multiple products with commercial value and can increase the profitability from the environmentally friendly polyculture systems compared to monoculture products [232].

The article "Advantage of Species Diversification to Facilitate Sustainable Development of Aquaculture Sector" was retracted in 2022. Reasons: plagiarism; overlap with other authors' work.

## 4. Future Implications

Indeed, no specific factors or criteria are responsible for turning aquaculture systems into ventures susceptible to failure. Reasonably, it can be a combination or set of variable factors that involve biological and ecological knowledge, management effects, and socio-economic parameters. Fisheries can be classified into three groups (fail, deplete, and sustainable); the overall ratings are in a wide range, suggesting wide diversity in terms of capacity and processes involved in fishery management [233]. Sustainable aquaculture features important factors, including productivity, resilience, conservation, economic viability, and environmental friendliness [234]. Therefore, evaluating the sustainability features of polyculture systems requires addressing several issues involved in aquatic farming. Furthermore, future aquacultures must be ethical, sensitive, and socially just. Besides this, there are growing concerns about the well-being of fish in aquaculture systems, as suggested in the “FishEthoBase” database [235], which must be appropriately enforced in future aquaculture systems.

Despite the existing COVID-19 pandemic’s prolonged negative impact on the global fish economy [236], the aquaculture industry can be expected to thrive and play a significantly important role in promoting socio-economic development [237]. This sector is expected to continue supporting rural stakeholders’ livelihoods in several developing countries [238]. There is a need for continuous innovations in aquaculture technology that can be validated as the best alternative to drive sustainable aquaculture development to address current constraints and challenges [239,240]. However, several marginal farmers who practice aquaculture in rural areas tend to practice traditional farming systems; thus, the adoption of innovative technologies is lagging [226]. Therefore, the objectives of future studies should be to recognize key socio-demographic factors involved in the decision-making process and constraints in the adoption of new technologies in aquaculture systems, embrace all-inclusive sustainability, and examine economic profitability [25].

Land-based closed recycling aquaculture systems (RAS) among aquaculture practices are gaining popularity to develop industrial-scale aquaculture factories, wherein effluent water gets treated before being returned to the system, thus profoundly reducing the dependency on external water supplies [241,242,243]. In addition to RAS, biofloc aquaculture technology is being identified and used for a diverse range of aquaculture species either in monoculture or polyculture practices [76,162,243,244]. Currently, industrial-scale RAS is setting up a full grow-out to offer several opportunities to increase production volume in nations that have already established fish farming and new opportunities for countries with limited options to perform intensive fish farming [245]. However, industrial development requires verification in system operations at different scales and intensities, which certainly involves higher financial risk until the aquaculture technologies and processes are well examined under given conditions [243]. There is a need for capital investment and government policy support in this stage. At present, numerous RAS technology providers are encountering these concerns, and intensive RAS aquaculture with non-sensitive species is prepared to enter the mainstream [50]. In merely technical terms, system operation at moderate stocking densities, with non-sensitive species, or at early life stages has succeeded with RAS technology, including for more sensitive fish species like salmonids [246]. As industrial aquaculture technologies are moved from the laboratory level to the phase of industrial use verification, economic risk shifts from capital associated with time expenses and prototype engineering at a small scale to the risks involved with investing in large-scale facilities. Furthermore, the likelihood of losing industrial-scale raising stock can be a costly scenario compared to investigating with small-scale batches of sensitive and non-sensitive fish species in prototype aquaculture systems. An important criterion to achieve success and rapid industrialization is careful planning of the core aquaculture technology in the early stage and considering independent production units to reduce and sort out economic risk, which aids in integrating the backbone of the autonomous RAS system.

The article "Advantage of Species Diversification to Facilitate Sustainable Development of Aquaculture Sector" was retracted in 2022. Reasons: plagiarism; overlap with other authors' work.

## 5. Conclusions

Aquaculture can be more diverse, with a range of species including fish, shellfish, crustaceans, mollusks, aquatic plants, and algal species cultivated globally in a wide diversity of marine, brackish, saltwater, and freshwater settings. It is pivotal to enforce sustainable aquaculture development from a socio-economic and environmental standpoint. Current aquaculture practices employ diverse species groups, locations, systems, resource utilization patterns, a wide range of diversification prospects, and other aspects. However, scientific and operational consensus about these alternative options to achieve more sustainability must still be reached. Exploring aquaculture approaches would facilitate environmental protection, human well-being, diversified income sources, and sustainability among aquaculture practices [247,248]. Polyculture practices involve combining a group of species based on multiple ecosystem functions and species that can share the given ecosystem with more positive interactions. Species compatibility among combined species is inevitable for successful polyculture practices. Thus, such systems require considering both species complementarity and compatibility simultaneously. Some combined fish species may be naturally compatible or have basic species compatibility, and the alternative is an intended species compatibility that can be facilitated via manual operations. The polyculture approach considers the combination of species to utilize a range of accessible resources (space, food, and shelter) under basic species complementarity or uses multiple components in IAA systems or via the advantages of mutualism or commensalism to achieve species compatibility and complementarity. The most preferred approach is polyculture to establish the most profitable and socially acceptable aquaculture practices, which considers integrated management and ensures sustainable development [249].

Polyculture practices in aquaculture have several positive aspects, including improved productivity, resource sharing, environmental protection, and animal welfare by leveraging agroecology principles and ecological functions based on aquaculture concepts. First, the polyculture approach promotes synergies among abiotic/biotic compartments, reinforces the efficient use of resources, and decreases carbon and ecological footprints. Second, the polyculture approach can improve the system resilience of aquaculture based on species diversity, which facilitates adaptation to varying ecological circumstances.

Third, such systems are appropriate for growing unprofitable species in monoculture or other high-value species depending on their trophic behavior, or alternatives to the conventional cleaning methods. The fourth significant aspect of polyculture is the need for increased social acceptance of products and ensuring animal welfare. However, more sustainable aquaculture development implies that well-trained growers understand the complexity of the polyculture systems, including spatiotemporal dynamics of biological and ecological processes.

## Figures and Tables

**Figure 1:** Schematic representation of aquaculture systems that involve basic complementarity. (**a**) Multi-trophic aquaculture involving unfed species based on the discrete trophic levels accessible in a farm setting, e.g., conventional aquaculture pond systems of carp species. (**b**) Mono-trophic aquaculture system involving two fed-fish species with the same trophic-level food resources (formulated feed pellets), e.g., open cage systems or RASs.

The article "Advantage of Species Diversification to Facilitate Sustainable Development of Aquaculture Sector" was retracted in 2022. Reasons: plagiarism; overlap with other authors' work.

**Figure 2:** Schematic illustration of aquaculture based on the principle of enhanced complementarity via trophic interactions amongst combined species. In IMTA, water flow supports the multi-trophic interactions. This principle enables the utilization of the waste of one aquaculture subsystem as a food source for another. For instance, finfish species are reared based on pellet feeding. Extractive shellfish species utilize dissolved organic matter, and seaweed extracts the inorganic content: feces and uneaten food consumed by detritivorous sea cucumber species.

**Figure 3:** Schematic representation of an aquaculture system based on enhanced species complementarity via trophic interactions among the farmed species. This system integrated agriculture–aquaculture associated with terrestrial farming units and aquaculture systems. Herein, nutrient recycling is systematized among farm components, including terrestrial crops, co-products, livestock feed, and nutrients for aquatic settings (zooplankton and phytoplankton) as reported in the previous report [37].

**Figure 4:** Graphical illustration of a polyculture system based on enhanced species complementarity through beneficial interactions amongst combined fish species. (**a**) Polyculture system based on commensalism, a positive interaction among fish species. The foraging behavior of one fish species enhances feed resource availability needed for another fish species by playing a role in the resuspension of nutrients accumulated at the sediment layer from the water column. (**b**) Polyculture system based on the principle of mutualism between fish species. Both the fish species benefit from being cultivated together, e.g., in cage systems. Here, a cleaner fish protects client fish by controlling sea lice as stated in the previous report [152].

**Figure 5:** Types of polyculture systems: (**a**) direct polyculture, (**b**) pond-cum-cage polyculture, and (**c**) sequential polyculture. Compatible species other than those shown in the figure can be cultured.

**Table 1:** List of glossary terms and aquaculture-related concepts used in the article.

Concept	Description	Reference
Agrochemicals	Chemicals used in agriculture including insecticides, fungicides, weedicides, growth promoters, and fertilizers. Agrochemical-based monoculture of aquatic species must be heavily opposed and stopped in the interest of human health and environmental protection.	[33]
Agroecology	The application of ecological principles to improve agricultural systems and practices leads to new farming methods that increase yield while reducing environmental impact.	[34]
Aquaponics	An aquaculture system that recycles waste produced by combined aquatic animals to provide nutrients for hydroponically grown vegetables and simultaneously purify the water.	[35,36]
Aquaculture	The breeding, rearing, and harvesting of aquatic animals or cultivation of aquatic plants for food; essentially, it means farming in water.	[37]
Biodiversity	A measure of variation at the genetic, taxonomic, species, and ecosystem levels.	[38]
Commensalism	A biological association between two animals, wherein one derives benefits and the other derives neither advantage nor harm.	[39]
Ecological engineering	The deliberate design of ecosystems to mutually benefit humans and nature.	[40]
Ecological footprint	The impact of an individual human or community directly on the environment; it is expressed as the amount of land area necessary to sustain given resources.	[41]
Ecological functions	Various organisms perform different positive ecological functions in a given ecosystem.	[42]
Ecological intensification	A knowledge-intensive procedure that involves the optimum functioning of environmental functions and biodiversity aspects to improve the overall performance of the agricultural system and eventually the farmers’ livelihoods.	[16]
Ecosystem services	The multitude of benefits that the ecosystem provides to human society. Biodiversity is essential to enforce ecosystem functions and the delivery of ecosystem services.	[43]
Facilitation	An ecological process categorized under commensalism interactions that refers to positive species interactions benefitting at least one species and causing harm to neither.	[44]
Integrated agriculture–aquaculture (IAA)	Combining two or more activities that involve agriculture, aquaculture, and household components.	[45]
Integrated multi-trophic aquaculture (IMTA)	A concept that harnesses the food chain, wherein the waste generated by one species nourishes another. This farming approach involves culturing a fed species in combination with an extractive species that can use the waste from the former as nourishment for their growth.	[46]
Monoculture	Farming a single species at any intensity, either in water or land.	[47]
Mutualism	A common type of positive ecological interaction that can be categorized into either facultative or obligate interactions, wherein both combined species derive overall benefits.	[39]
Polyculture	Sustainable agriculture approach that involves the simultaneous culture of several species in one location based on the ecological principle of species diversity designed by imitating natural ecosystems.	[48]
Recirculated aquaculture system (RAS)	An indoor aquaculture system that purifies and recirculates the same water. It has a low footprint and allows safe year-round farming under controlled conditions.	[49,50]
Resilience	In an ecological context, resilience is the ability of an ecosystem to overcome disturbances or stresses by reorganizing to maintain normal functioning while undergoing changes.	[51]
Species diversity	Overview of the number of different species that coexist in an ecosystem and their relative abundances.	[24]
Species compatibility	A phenomenon wherein combined taxa can co-exist in the same ecosystem without negative or detrimental interactions (predation, parasitism) or competition for resources (space, food, or shelter).	[52]
Species complementarity	The capacity of a combined species to utilize different parts of accessible resources that include by-products of combined species, or their capacity to exhibit positive interactions (either mutualistic/commensal) and contribute to the sustainability of the aquaculture systems.	[52]
Sustainability	Achieving economic, ecological, social, and human needs without compromising the loss of essential resources required for future generations.	[14]

The article "Advantage of Species Diversification to Facilitate Sustainable Development of Aquaculture Sector" was retracted in 2022. Reasons: plagiarism; overlap with other authors' work.

**Table 2:** Illustration of case studies published on polyculture and integrated aquaculture systems that ensure improvement of ecological sustainability as well as social and economic development (ethical, socially just, local food security, and diversified income). It can be categorized into two types: (a) basic complementarity, where the combination of compatible species facilitates the utilization of different accessible resources (feed, space, or shelter), and (b) enhanced complementarity, where combined species utilize co-products of another taxa/species, exemplifying aquaculture systems such as IMTA, IAA, and advantages of mutual or commensal relationships. Recirculated aquaculture system (RAS).

Aquaculture Case Studies	Consequences for Sustainability	Process Implications	References
**Basic Complementarity**			
Polyculture of juvenile pikeperch fish and sterlet fish in an RAS.	Requires less labor than that required to grow the same species in monoculture systems.	Benthic trophic behavior of starlet fish allows them to use food that accumulates at the bottom.	[63]
Polyculture system study effect of behavior on the production of pikeperch in an RAS.	Upgrades production performance, increasing mass from 25 to 51% compared to that in a monoculture system.	Improves spatial resource use and decreases competition for trophic resources among combined fish species.	[76]
Freshwater aquaculture of fish species in cage systems ensures the consumption of non-consumed food dispersed in the internal cages.	Maintains water quality without risk of the fish escaping. Suitable for exotic farm species.	Polyculture system for fish in multi-layered cages, suitable for high-value sturgeon (*Acipenser* sp.) in the internal cage area and cyprinids (silver carp (*Hypophthalmichthys molitrix*) and bighead carp (*Hypophthalmichthys nobilis*), and in the external cages considering crucian carp (*Carassius auratus*)).	[72]
**Enhanced Complementarity**			
The IMTA system: farming of pellet-fed aquaculture species, e.g., shrimp or fish species whose extracts dissolve organic or particulate matter, e.g., fish, mollusks, and echinoderms; extracts or dissolved organic–inorganic matter is feed for species e.g., microorganisms, macrophytes, and macro-algae.	Maintains water quality and improves nutrient cycling within IMTA systems. Improves diversification of production: About 50% of feed proteins are converted into consumable protein.	Combines several species based on ecological functionality.	[46]
IMTA system: intensive and semi-intensive aquaculture system: prawn (*Macrobrachium amazonicum*) and tilapia (*Oreochromis niloticus*).	Helps to improve nutrient cycling and diversification of aquatic food products.	Combines several species based on ecological functionality that ensures that co-products of one species function as a feed source for the other.	[77]
IMTA system: iliophagus (*Prochilodus lineatus*) integrated with benthic shrimp (*Macrobrachium amazonicum*) and pelagic fish (*Colossoma macropomum*).	Helps improve nutrient cycling in aquaculture ponds because the waste of one species is a valuable feed for the other species. It also helps improve diversification production by increasing total species yields by about 35%.	Combining fed fish species with two other fish species fed on the wasted feed and waste of another species.	[78]
IMTA system: involves the aquaculture of fish (*Sebastes schlegeli*), shellfish (*Haliotis discus hannai*), and sea cucumber (*Apostichopus japonicas*) in an RAS.	This system helps improve nutrient cycling. Aquaculture of shellfish and sea cucumber is also known to improve nitrogen and phosphate budgets. It improves diversification and increases the growth rate compared to those of monoculture systems.	Combining different species in aquaculture based on their diverse feeding habits and ecological niches, e.g., pellet-fed species with deposit-fed species.	[79]
IMTA system: a combination of several plant species, e.g., water lettuce (*Pistia* spp.), water convolvulus (*Ipomea aquatica*), and water hyacinth (*Eichhornia crassipes*) along with combined fish, e.g., grass carp (*Ctenopharyngodon idella*) or shellfish species.	Helps maintain the water quality. The plant species are involved in removing total nitrogen and total phosphorus while decreasing chemical oxygen demand. This system increases the yield of grass carp, improves survival rate, and reduces drug use compared to conventional aquaculture systems run without aquatic plant species. Production of value-added products (salads, vegetables).	In addition to their enhanced water purification efficiency, plants consume nutrients released by fish or shellfish species. Microbes that grow on the roots of plants degrade pollutants and reduce excess nutrients dissolved in water (N and P). Plants also provide natural habitats for fish and shellfish species.	[40,80]
**Integrated Agriculture–Aquaculture (IAA)**			
IAA system: maintaining the diversity of integrated rice and fish production.	Improves diversification of farm products and increases economic feasibility.	Combines several species and maintains diversity based on ecological functioning.	[33]
IAA system: using waste from livestock and other agricultural practices to fertilize fishponds. Applying fishpond sediments to fertilize agricultural land. Using by-products of the crop to feed livestock (cattle, poultry, and pigs) and combined fish species.	Helps recycle nutrients from terrestrial agricultural systems to aquaculture systems and vice versa, either directly or indirectly. Helps increase the yield of livestock and aquaculture.	Combines several species based on their ecological functions.	[55,81]
IAA system: integrating terrestrial rice farming with freshwater prawn (*Macrobrachium rosenbergii*).	Improves diversification of production and increases economic feasibility.	The IAA system is multi-spatial and utilizes both water and soil resource utilization more efficiently than monoculture systems.	[82]
**Commensal Relationship**			
Commensal relationship: Combines carp (*Cyprinus carpio*) and rohu (*Labeo rohita*) in a pond.	Increases productivity by approximately 40% compared to rohu monoculture.	Facilitation relationship: redispersion of feed by the carp species.	[83]
Commensal relationship: polyculture of omnivorous fish (*Takifugu obscurus*) and white shrimp (*Litopenaeus vannamei*).	Increases productivity owing to better animal welfare and health conditions. Improves the resistance of shrimp species and protects them against diseases. Improves the survival rate of shrimp species.	Antibacterial and antifungal properties of fish mucus improve the survival rate of white shrimp species.	[84]
Commensal relationship: Between jellyfish and juvenile carangids in coral reef habitats.	Protects juvenile carangids from predators because they hide in the vicinity of jellyfish tentacles that are used as a shield against potential predators.	The coral reef habitat facilitates the commensal relationship between juvenile carangid and jellyfish, allowing carangid fish to sustain their stock.	[85]
Commensal relationship: polyculture of grey mullet (*Mugil cephalus*) with white shrimp (*Litopenaeus vannamei*).	Improves farm performance and water quality. Decreases parasite attacks in polyculture because of low amounts of total organic matter and sediments in the water.	Involves species that improve the quality of the farm environment due to their commensal feeding behavior and diet habits.	[86]
Mutualism: polyculture system for cleaner shrimp (*Lysmata vittata*) and orange-spotted grouper (*Epinephelus coioides*).	Ensures environmental protection because combining these species in culture is a safer alternative than using chemical treatments for parasitic diseases. It also helps to improve diversification of production, thereby increasing economic feasibility. Cleaner shrimp species have high-value ornamental purposes. This species feeds on fish parasites.	Involves species that act as natural predators by feeding on parasites and other pathogens. It provides a safe alternative to chemical treatment.	[87]

The article "Advantage of Species Diversification to Facilitate Sustainable Development of Aquaculture Sector" was retracted in 2022. Reasons: plagiarism; overlap with other authors' work.

## Data Availability

Not applicable.
